RETRACTED

# Progress of Noncoding RNA Regulating the Growth and Development of Antler Tissue Research

**DOI:** 10.1155/2022/3541577

**Published:** 2022-07-19

**Authors:** Yipu Wang, Wei Hu

**Affiliations:** Biochemistry and Molecular Biology, Jilin Agricultural University, Changchun City, Jilin Province 130000, China

## Abstract

Antler is the secondary sexual characteristic of deer, which develops on the forehead at puberty. It is the only organ that can be regenerated entirely in mammals. Therefore, it is often used as a research model in the field of organ regeneration and wound repair. Many growth factors and proteins play an active role throughout the developmental process of antler regeneration. With the rapid development of sequencing technology, more and more noncoding RNAs (ncRNAs) have been discovered, and the relationship between ncRNA and antler regeneration has gradually become clear. This paper focuses on the research progress of several ncRNAs (including miRNA and lncRNA) in deer antler tissues, which are helpful to reveal the molecular mechanism of deer antler regeneration at the molecular level.

## 1. Introduction

Sika deer (*Cervus nippon*), alias Hua Lu, belongs to the genus Artiodactyl in animal taxonomy. China is one of the countries with the most abundant deer resources in the world. Antler is the horn of unossified dense antler, which attracts the attention of many scholars, depending on the unprecedented growth rate, regeneration mechanism, and fantastic medicinal value of other animal organs. It is also the only organ that can be regenerated in mammals [1]. The growth of antler depends on the formation of the pedicle. The occurrence of the pedicle is closely related to the antiresistance periosteum (AP) on the lateral crest of the frontal bone of the deer [2]. The pedicle is formed by the further proliferation and differentiation of AP under the action of testosterone during puberty and then develops into antler [3]. In autumn, antler growth entirely and begins to ossify, and the velvet begins to fall off. The ossified antlers will fall off naturally after the next spring. The rapid healing of the wound on the pedicle indicates the beginning of a new round of regeneration of antler [4]. Meanwhile, every regeneration of antler is based on pedicle periosteum (PP). After the loss of the ossified antlers the previous year, PP facilitated the wound healing at the broken antlers. PP proliferates and differentiates further at the wound to form a new antler [5–7].

The antler can grow as 1.14 cm/d, which is faster than the proliferation of cancer cells, and the velvet antler tissue formed under such a rapid growth condition does not show any signs of cancer. Therefore, many scholars believe that the rapid growth of antler has a unique material basis. With the further study of antler, it has been found that the growth of antler is regulated by a variety of specific molecular mechanisms. A variety of cell growth factors and hormones play an essential role in promoting the growth of antler and promoting the proliferation and differentiation of antler cells. For example, insulin-like growth factor (IGF), transforming growth factor (TGF), epidermal growth factor (EGF), nerve growth factor (NGF), androgen and growth hormone, and so forth[6–8]. The autocrine and paracrine stimulation of a variety of growth factors is crucial for the rapid proliferation of antler growth tissue. In the process of tissue repair, growth factors can increase cell mitotic activity and promote the transformation of cell cycle or promote the synthesis of nucleic acid, protein, and other cellular components [9–12].

RETRACTED

Deer antler regenerates every year, providing a good model for regenerative medicine research. Deer antler cartilage is a very unique cartilage tissue, and the uniqueness of deer antler makes it an important model for the study of cartilage regeneration and repair mechanisms. In addition, deer antler cells proliferate rapidly in a period of rapid growth without canceration, making them an important model for cancer treatment research. However, the regulatory mechanism of the rapid proliferation of deer antler stem cells without canceration is still unclear, and its research is of great significance. Therefore, this study is aimed at summarizing the research status of noncoding RNA regulation of velvet antler tissue growth and development and at providing theoretical basis for velvet antler researchers.

## 2. Research Progress of miRNA Regulating the Growth and Development of Antler Tissue

### 2.1. Biosynthesis and Function of miRNA

In 1993, Lee et al. discovered miRNA (lin-4) in nematodes for the first time and confirmed that as a posttranscriptional regulator, it plays an important role in the regulation of gene expression through complete or incomplete complementary pairing with the 3′UTR of the target mRNA [13]. Subsequently, the existence of miRNA was found in various organisms, and the transcription of RNA can be regulated by specific binding to mRNA [14]. miRNA is a kind of noncoding RNA (ncRNA) with high conservatism and tissue specificity. It has extraordinary structural features, generally with a length of 21-23 nt and often with a hairpin structure. The DNA that encodes miRNA in organisms is often strung together to form a miRNA gene cluster. Per-miRNA, with polynucleotide tail and cap structure, was formed under the cleavage of RNase II and then cut into small segments of double-stranded RNA, under the action of Drosha RNase. Finally, one strand of double-stranded RNA was degraded, and the other single strand of RNA was mature miRNA [15, 16]. After the mature miRNA binds to the Ago protein, the RNA-induced silencing complex (RISC) is formed and then inhibits or silences the target gene by binding to the three-prime untranslated regions (3′UTRs) on the target mRNA. According to the literature, more than half of mRNA is regulated by miRNA, which is one of the main functions of miRNA in organisms [17]. Interestingly, the regulation of miRNA and mRNA is not a corresponding one-to-one relationship. Sometimes an miRNA may act on multiple mRNAs, and the same mRNA may be regulated by multiple miRNAs [18, 19].

RETRACTED

In recent years, more and more literature has reported that the differential expression of the same kind of miRNA has been found in the growth and development processes of many organisms [20, 21]. This also makes people wonder whether these miRNAs regulate the growth and development of organisms by downregulating the expression of proteins encoded by self-binding mRNA. As a result, more and more miRNA, which plays an important regulatory role, has been found that the differential expression of miRNA in different developmental stages of the same tissue is of great significance in the study of its growth and development mechanism [22, 23].

### 2.2. The Role of miRNA in the Growth and Development of Antler

The antler is a natural library of cell growth factors. Insulin-like growth factor (IGF) [24, 25], vascular endothelial growth factor (VEGF), and transforming growth factor (TGF) have been found in the apical tissue of antler. The growth of antler includes the process of antler skin growth, vascular extension, mesenchymal development, cartilage growth, and so forth. These growth factors are involved in each growth process and participate in the regeneration of antlers. Therefore, the growth process of antler is regulated by a variety of growth factors. The study on the regulation mechanism of growth factors in the tissue of antlers will provide a robust basis and some new ideas for exploring the mechanism of the complete regeneration of antlers.

#### 2.2.1. Expression Pattern of miRNA in Antler Tissue

At first, Hu et al. [26–28] constructed an miRNA microarray of antler apical cartilage and mesenchymal tissue and analyzed the differential expression of miRNA. A total of 289 miRNA, miRNAs were found in the mesenchymal layer, and 304 miRNAs were found in the cartilage layer. There were 158 differentially expressed miRNA between two different tissues. According to Ba et al. [29], next-generation sequencing technology was used to sequence miRNA in two different regions of pedicle periosteal stem cells. A total of 20 conserved and specific miRNA sequences were found. Furthermore, the results of miRNA sequencing were divided into 167 miRNA families, of which miR-296 was specific to embryonic stem cells. During the growth of antler, the expression level of 8 miRNA decreased, and 6 miRNAs increased. Through GO biology process analysis, it was found that these miRNAs were involved in the regulation of Wnt [30], MAPK [31], and TGF-*β* [32, 33] signaling pathways related to tissue growth and regeneration.

RETRACTED

Han et al. [34] carried out the HiSeq deep sequencing of antler apical cartilage and mesenchymal tissues. The obtained siRNA was screened to remove the sequences with poor quality and length less than 18 nt, and then, the screened results were analyzed. The results showed that there were 25415291 small RNA and 122112 species in antler cartilage and mesenchymal tissues. The specific sequences of chondrocytes and mesenchymal cells were 363590 and 439528, respectively. The specific sequences of mesenchymal cells were 466685 and 578253, respectively. The differential expression of the known miRNA in the sequencing results was analyzed. Among them, 743 upregulated miRNA and 147 downregulated miRNA were found in chondrocytes, and the same miRNA regulation was found in mesenchymal cells as in chondrocytes, with 785 upregulated and 157 downregulated, respectively. The number of miRNAs with a significant difference in two different kinds of cells was 666. These results confirm that there are many differentially expressed miRNA during mesenchymal chondrogenic differentiation. These miRNAs may affect the expression of their target genes and regulate the process of antler regeneration by combining with their specific target genes, which also lays a foundation for the study of deer miRNA.

#### 2.2.2. Regulation of IGF Signal Pathway by miRNA

IGF is a kind of multifunctional regulatory factors of cell proliferation, which is named because its chemical structure is similar to that of insulin [35]. IGF plays a significant regulatory role in cell growth and embryonic development. Many literatures have reported that VEGF and its receptor EGFR are highly expressed in velvet antler tissue and participate in the growth and regeneration of velvet antler tissue [36, 37].

In our early study, Hu et al. [26–28] synthesized four pairs of pre-miRNA precursor fragments according to the mRNA sequence of IGF-1 and transferred them into the eukaryotic expression vector to construct recombinant plasmids and transfect antler tissue cells. The results showed that after transfection of IGF-1 recombinant plasmid, the expression level of IGF1 mRNA and IGF1 protein in antler chondrocytes decreased, the proliferation of chondrocytes in vitro was inhibited, the percentage of cells in the S phase of the cell cycle decreased, and the growth cycle was stagnated in G0/G1 phase. The results showed that the expression level of IGF-1 was regulated by related miRNA.

RETRACTED

Hu et al. [38] further studied and found. In miRNA GeneChip, 126 miRNAs were upregulated, and 84 miRNAs were downregulated in cartilage. The miRNA that can combine with the 3′UTR of IGF-1 is predicted by using the TargetScan Human software. miR-1 was selected for next experiment, miR-1 mimic was designed, and it was transfected into antler chondrocytes to make it overexpressed in chondrocytes. The targeting relationship between miR-1 and IGF-1 was verified by a double luciferase reporting experiment. Then, fluorescent quantitative PCR and Western blot experiments were used to verify the regulation of miR-1 on IGF-1. The results showed that miR-1 could downregulate the expression of IGF-1 protein in antler chondrocytes.

Hu et al. [26–28] used the TargetScan bioinformatics software to screen out miRNA that can combine with IGF-1R and exert its function. The results showed that let-7a and let-7f could bind to IGF-1R, and IGF-1R was one of the target genes of let-7a and let-7f. Quantitative real-time PCR showed that the expression of let-7a and let-7f mimics in antler chondrocytes increased significantly at 24 h, 48 h, and 72 h after transfection. Cell proliferation was detected by the MTT method, and the cell cycle structure was detected by flow cytometry. The results showed that let-7a and let-7f mimics had a constant effect on the proliferation of antler chondrocytes. The percentage of S phase cells decreased. Western blotting results showed that the expression of IGF-1R decreased after the transfection of let-7a and let-7f mimics, while the expression of IGF-1R increased after the transfection of let-7a and let-7f inhibitor.

#### 2.2.3. Regulation of VEGF Signal Pathway by miRNA

According to the literature, vascular endothelial growth factor (VEGF) plays a vital role in the growth of antler [26–28, 39, 40]. VEGF acts on vascular endothelial cells; it acts as a mitogen to promote vascular endothelial cell division and proliferation [41, 42], hematopoietic stem cells, and venules explicitly. At the same time, studies have shown that VEGF plays a particular role in inducing angiogenesis and enhancing capillary permeability [43, 44]. It specifically binds to the receptors on the surface of vascular endothelial cells, stimulates the continuous proliferation of vascular endothelial cells, and participates in the regulation of vascular cell formation in physiological and pathological processes [45].

RETRACTED

Li et al. (Li [46]), using bioinformatics analysis methods, preliminarily screened the miRNA related to the regulation of VEGF in the miRNA microarray of antler apical cartilage and mesenchymal tissue. The screening results showed that 8 miRNAs associated with VEGF and differentially expressed were found in the microarray. Further screening by SYBR Green real-time quantitative real-time PCR and Western blotting techniques showed that miRNA-93-5p and miRNA-20b-5p could specifically bind to VEGF 3′UTR sequence, and the expression level was the highest, and the inhibition effect of VEGF protein expression level was the most obvious after transfection of miRNA-93-5p and miRNA-20b-5p. The results of the double luciferase experiment showed that miRNA-93-5p and miRNA-20b-5p could regulate the VEGF gene, and VEGF was the target gene regulated by miRNA-93-5p and miRNA-20b-5p. In order to further study the regulation of the VEGF gene by miRNA-93-5p and miRNA-20b-5p, the authors transfected miR-93-5p and miR-20b-5p into antler chondrocytes and detected them by Real-time quantitative PCR after 24 h, 48 h, and 72 h culture. The results showed that miR-93-5p and miR-20b-5p were highly expressed in antler chondrocytes. After transfecting antler chondrocytes with miR-93-5p and miR-20b-5p in vitro, it was found that the proliferation of antler chondrocytes was significantly inhibited, and the expression level of VEGF protein continued to decrease with time. In summary, it can be concluded that miR-93-5p and miR-20b-5p may affect the expression of VEGF protein by regulating VEGF in antler chondrocytes, thus regulating the growth and development of antler.

VEGF can induce micro angiogenesis and enhance vascular permeability by binding to its receptor (VEGFR) to participate in the regulation of biological processes such as endothelial cell growth. We have confirmed that there are related miRNAs in antler chondrocytes that can regulate the expression of VEGF, but are there also miRNAs that directly regulate VEGFR involved in regulating the growth and development of antler cartilage?

With such a scientific question, Liu et al. [47] screened two miRNAs, miRNA-15a, and miRNA-15b, which can bind to VEGFR and differentially expressed in antler apical tissue miRNA microarray. Fluorescent quantitative PCR showed that miRNA-15a and miRNA-15b were highly expressed in antler cells, and the level of VEGFR decreased in the transfected antler cells, which may be related to the inhibition of the proliferation of the cells in vitro. The experimental results of Li and Cui confirmed the existence of miRNA in antler cartilage and regulated the growth and development of antler by combining with target genes.

RETRACTED

#### 2.2.4. Regulation of TGF-*β* Signal Pathway by miRNA

In addition to VEGF, the special biological process of antler chondrocytes is also inseparable from the regulation of a large number of growth factors. According to the literature, the apical tissue of antler contains the expression of many growth factors, including TGF-*β*1 and TGF-*β*2[48], among which TGF-*β* is one of the many growth factors. TGF-*β* has many biological functions, such as cell proliferation, differentiation, apoptosis, and embryogenesis (A. [49]). It also plays a certain role in the formation of cartilage. Many literatures have reported that TGF-*β* is highly expressed in antler chondrocytes and participates in the proliferation and differentiation of antler chondrocytes [50–52].

So is there a noncoding factor in the TGF-*β* signal pathway that regulates the protein molecules of the TGF-*β* superfamily? There are a large number of conserved gene clusters in vertebrate genes, each of which has a clear division of labor, and each gene cluster has its own family members, and current studies have shown that the miRNA-17-92 gene cluster has an important impact on the TGF-*β* pathway. Yan et al. [53] analyzed the members of the miRNA-17-92 gene cluster and screened two members of the miRNA-17-92 gene cluster, namely, miRNA-19a and miRNA-19b, which were significantly differentially expressed against sika deer TGF-*β*RII. Further research on the proliferation law of antler chondrocytes showed that TGF-*β*RII is a target gene that regulates key miRNAs in this process. After transfection of miRNA, the expression level of target gene proteins was inhibited.

Han et al. [34] screened six differentially expressed miRNAs. The most differentially expressed miRNA was verified by deep sequencing, and the results showed that TGF-*β*2 was a target gene regulated by miRNA-148a-3p. At the same time, the proliferation of antler chondrocytes was inhibited after miRNA-148a-3p transfection, and the relative expression levels of TGF-*β*2 protein and related proteins TGF-*β*RII and IGF-1 were also decreased.

Liu et al. [54] verified differentially expressed miRNA in antler cartilage and mesenchymal tissues by quantitative real-time PCR, in which the expression levels of miRNA-18a and miRNA-106b were the highest. Double luciferase activity assay confirmed that there were binding sites of miRNA-18a and miRNA-106b in 3′UTR of Smad2 and Smad4. Smad2 is a target gene regulated by miRNA-18a, and Smad4 is a target gene regulated by miRNA-106b. According to the experimental results, it can be known that the normal proliferation process of chondrocytes is inhibited by the regulation of Smad2, and the relative expression levels of Smad2 protein and related proteins TGF-*β*1 and TGF-*β*2 decreased in a time-dependent manner, while the relative expression levels of Smad4 and Smad6 increased and Smad1 decreased after transfection of miRNA-106b. These results further indicate that the IGF, VEGF, and TGF-*β* signal pathways of sika deer are closely related to miRNA, and the growth process of antler is regulated by miRNA.

RETRACTED

## 3. Research Progress of lncRNA Regulating the Growth and Development of Antler Tissue

### 3.1. lncRNA and Its Biological Function

Long noncoding RNA (lncRNA) is a non-protein-coding RNA transcript with a length of more than 200 nt [55]. Because of its extraordinary length, lncRNA is relatively less conservative and stable compared with other kinds of noncoding RNA. Therefore, at first, lncRNA was regarded by researchers as a transcriptional by-product of Poly II without any biological function [56]. However, with the in-depth research of transcriptome, more and more literature has reported that lncRNA is involved in the development of a variety of biological processes and gene expression regulation in vivo [57]. Scientists pay more and more attention to the related research of lncRNA. The biological functions of lncRNA include regulating gene expression by regulating DNA/RNA methylation and demethylation, combining with transcription factors or participating in transcriptional regulation as transcription factors, participating in posttranscriptional regulation in variable splicing and editing of mRNA, acting as the precursor of small RNA such as miRNA and piRNA, and acting as a sponge to combine with specific miRNA to regulate the expression of target genes by controlling the expression of miRNA[58, 59].

### 3.2. The Role of lncRNA in the Growth and Development of Antler

Chen et al. [60] carried out high-throughput sequencing of antler mesenchymal and cartilage tissues to detect the changes of lncRNA expression between two different tissues and then analyzed the target gene of lncRNA by bioinformatics techniques. lncRNA and mRNA related to antler regeneration were screened out. An lncRNA-mRNA interaction network diagram related to osteogenic differentiation, cell proliferation, and migration was constructed. Its accuracy was verified by real-time quantitative PCR. The results showed that four target genes related to bone formation were found. They were simultaneously regulated by 5 lncRNAs and found 2 target genes related to cell proliferation, which were coregulated by 8 lncRNAs and 3 target genes related to migration, and they were coregulated by 4 lncRNAs. The results of quantitative real-time PCR were consistent with those of high-throughput sequencing. It can be verified. The lncRNA mentioned in the above experiments may regulate the regeneration process of antler by regulating functional target proteins such as bone formation, cell proliferation, and cell migration, so as to accelerate the regeneration and development of antler.

RETRACTED

Han et al. [61] carried out high-throughput transcriptome sequencing of the apical mesenchymal tissue of antler in three different growth periods (30 d, 60 d, 90 d). The expression differences of noncoding RNA (lncRNA; miRNA) in three different growth stages were analyzed, and the differentially expressed genes, by GO and KEGG enrichment analysis. Finally, the ceRNA network of RNA in the apical mesenchymal tissue of antler was constructed. The results showed that there were a large number of differentially expressed noncoding RNA in mesenchymal tissues of three different stages. The results of GO enrichment analysis showed that these differential RNAs were enriched in cell development, tissue development, phylogeny, and animal organ development. The results of KEGG enrichment analysis showed that these differentially expressed RNA, cGMP/PKG, and PI3K/AKT were related to growth, development, and cell cycle-related signal pathways. Combined with the results of enrichment analysis, the ceRNA network related to antler development was constructed. The results of these lncRNA studies of antler tissue enrich the study of noncoding RNA in Cervidae. It also further proved the molecular regulation of noncoding RNA on the regeneration and development of antler.

## 4. Discussion

Nowadays, the related studies of miRNA, lncRNA, and other noncoding RNA are often used to compare the expression differences between normal and diseased tissues at different developmental stages and to explore the process of tissue development and disease development from the perspective of endogenous competitive RNA or noncoding RNA. Because of its unique growth cycle and growth rate, antler has been used by researchers at home and abroad as a related research model in the fields of amputated limb regeneration, organ injury repair, and so forth. The process of antler regeneration is inseparable from the continuous transformation of mesenchymal cells to chondrocytes. These rapid proliferation and transformation seem to have some similarities with the occurrence and development of some diseases such as cancer. Therefore, we believe that the study of noncoding RNA in the apical tissue of pilose antler will be of great help to solve the mystery of the rapid growth of antler.

RETRACTED

Through the regulation of TGF-*β*, VEGF, and IGF signaling pathways, miRNA makes TGF-*β*1 differentially expressed in different parts of the antler tip, maintains the rapid proliferation of antler chondrocytes and inhibits its premature ossification, and regulates the rapid growth of velvet antler without canceration. VEGF may stimulate the rapid formation of blood vessels and participate in the regulation of bone calcification, resorption, and reconstruction. The division and proliferation of antler stem cells are proportional to the concentration of IGF-1, which can promote the proliferation of antler mesenchymal cells. But the regeneration of deer antler is a complex process involving many tissues, growth factors, hormones, and other factors [62]. The specific control mechanism still needs to be further explored. The discovery of miRNAs that regulate related transforming factor signaling pathways provides new ideas for studying the mechanism of deer antler regeneration.

The results of high-throughput sequencing of apical antler tissue also showed that there were differentially expressed lncRNA in mesenchymal cells and chondrocytes, as well as in mesenchymal cells at different growth and development stages. As a very special length noncoding RNA, lncRNA regulates target genes in many ways, although it is less conservative and stable than other kinds of noncoding RNA. Our study shows that there is an lncRNA in the apical tissue of antler, which can regulate its corresponding target genes, which promotes the study of noncoding RNA in the apical tissue of antler. In previous studies, people mostly predicted and screened some specific factor-related regulatory miRNA, but there are few reports about lncRNA as an miRNA molecular sponge to regulate target genes by competing with target genes to bind miRNA. The ceRNA network construction of the apical tissue of antler provides a reliable basis for later research. At present, the related research on circRNA only stays in the analysis and detection stage, and its circular structure and function verification still need to be identified and authenticated. In a word, the deepening and development of noncoding RNA in antler tissue will provide a new way to reveal the molecular mechanism of its regeneration and development.

Although deer antler can provide a basis for the treatment and research of various diseases, the regulatory mechanism of deer antler regeneration and rapid growth is still unclear. The internal regulation mechanism of deer antler is also very complex, and the specific mechanism still needs to be further explored so that it can be applied to real life more quickly.

RETRACTED

## Data Availability

The datasets used and analyzed during the current study are available from the corresponding author upon reasonable request.

## References

[1] Li C., Zhao H., Liu Z., McMahon C. (2014). Deer antler--a novel model for studying organ regeneration in mammals. *The International Journal of Biochemistry & Cell Biology*.

[2] Wang D., Berg D., Ba H., Sun H., Wang Z., Li C. (2019). Deer antler stem cells are a novel type of cells that sustain full regeneration of a mammalian organ-deer antler. *Cell Death & Disease*.

[3] Li C., Suttie J. M. (2003). Histological studies of bone formation during pedicle restoration and early antler regeneration in roe deer and fallow deer. *The Anatomical Record. Part A, Discoveries in Molecular, Cellular, and Evolutionary Biology*.

[4] Li C., Suttie J. M. (2001). Deer antlerogenic periosteum: a piece of postnatally retained embryonic tissue?. *Anat Embryol*.

[5] Li C., Suttie J. M., Clark D. E. (2005). Histological examination of antler regeneration in red deer (Cervus elaphus). *The Anatomical Record. Part A, Discoveries in Molecular, Cellular, and Evolutionary Biology*.

[6] Landete-Castillejos T., Currey J. D., Estevez J. A., Gaspar-López E., Garcia A., Gallego L. (2007). Influence of physiological effort of growth and chemical composition on antler bone mechanical properties. *Bone*.

[7] Li C. (2013). Histogenetic aspects of deer antler development. *Frontiers in Bioscience*.

[8] Pita-Thomas W., Nieto-Sampedro M., Maza R. M., Nieto-Diaz M. (2010). Factors promoting neurite outgrowth during deer antler regeneration. *Journal of Neuroscience Research*.

[9] Li C., Mackintosh C. G., Martin S. K., Clark D. E. (2007). Identification of key tissue type for antler regeneration through pedicle periosteum deletion. *Cell and Tissue Research*.

[10] Gaarenstroom T., Hill C. S. (2014). TGF-*β* signaling to chromatin: how Smads regulate transcription during self-renewal and differentiation. *Seminars in Cell & Developmental Biology*.

[11] Jones J. I., Clemmons D. R. (1995). Insulin-like growth factors and their binding proteins: biological actions. *Endocrine Reviews*.

[12] Iacovelli R., Sternberg C. N., Porta C. (2015). Inhibition of the VEGF/VEGFR pathway improves survival in advanced kidney cancer: a systematic review and meta-analysis. *Current Drug Targets*.

[13] Lee R. C., Feinbaum R. L., Ambros V. (1993). The C. elegans heterochronic gene lin-4 encodes small RNAs with antisense complementarity to lin-14. *Cell*.

[14] Ambros V. (2004). The functions of animal microRNAs. *Nature*.

[15] Nolte-'t Hoen E. N., Van Rooij E., Bushell M. (2015). The role of microRNA in nutritional control. *Journal of Internal Medicine*.

RETRACTED

[16] Wilczynska A., Bushell M. (2015). The complexity of miRNA-mediated repression. *Cell Death and Differentiation*.

[17] O'Connell R. M., Rao D. S., Chaudhuri A. A., Baltimore D. (2010). Physiological and pathological roles for microRNAs in the immune system. *Nature Reviews. Immunology*.

[18] Bartel D. P. (2004). MicroRNAs. *Cell*.

[19] Vishnoi A., Rani S. (2017). miRNA biogenesis and regulation of diseases: an overview. *Methods in Molecular Biology*.

[20] Wyman S. K., Parkin R. K., Mitchell P. S. (2009). Repertoire of microRNAs in epithelial ovarian cancer as determined by next generation sequencing of small RNA cDNA libraries. *PLoS ONE*.

[21] Nygaard S., Jacobsen A., Lindow M. (2009). Iden-tification and analysis of miRNAs in human breast cancer and teratoma samples using deep sequencing. *BMC Medical Genomics*.

[22] Rathjen T., Pais H., Sweetman D., Moulton V., Munsterberg A., Dalmay T. (2009). High throughput sequencing of microRNAs in chicken somites. *FEBS Letters*.

[23] Lagos-Quintana M., Rauhut R., Yalcin A., Meyer J., Lendeckel W., Tuschl T. (2002). Identification of tissue-specific mi-croRNAs from mouse. *Current Biology*.

[24] Suttie J. M., White R. G., Breier B. H., Gluckman P. D. (1991). Photoperiod associated changes in insulin-like growth factor-I in reindeer. *Endocrinology*.

[25] Suttie J. M., Gluckman P. D., Butler J. H., Fennessy P. F., Corson I. D., Laas F. J. (1985). Insulin-like growth factor 1 (IGF-1) antler-stimulating hormone?. *Endocrinology*.

[26] Hu W., Li T., Hu R., Wu L., Li M., Meng X. (2014). MicroRNA let-7a and let-7f as novel regulatory factors of the sika deer (Cervus nippon) IGF-1R gene. *Growth Factors*.

[27] Hu W., Meng X., Lu T. (2013). MicroRNA-1 inhibits the proliferation of chinese sika deer-derived cartilage cells by binding to the 3’-untranslated region of IGF-1. *Molecular Medicine Reports*.

[28] Hu W., Li T., Wu L., Li M., Meng X. (2014). Identification of microRNA-18a as a novel regulator of the insulin-like growth factor-1 in the proliferation and regeneration of deer antler. *Biotechnology Letters*.

[29] Ba H., Wang D., Li C. (2016). MicroRNA profiling of antler stem cells in potentiated and dormant states and their potential roles in antler regeneration. *Molecular Genetics and Genomics*.

[30] Mount J. G., Muzylak M., Allen S., Althnaian T., McGonnell I. M., Price J. S. (2006). Evidence that the canonical Wnt signalling pathway regu-lates deer antler regeneration. *Developmental Dynamics*.

[31] Zhang Y., Pizzute T., Pei M. (2014). A review of crosstalk between MAPK and Wnt signals and its impact on cartilage regeneration. *Cell and Tissue Research*.

RETRACTED

[32] Diao H., Wang J., Shen C. (2009). Improved cartilage regeneration utilizing mesenchymal stem cells in TGF-beta1 gene-activated scaffolds. *Tissue Engineering. Part A*.

[33] Yin F., Cai J., Zen W. (2015). Cartilage regeneration of adipose-derived stem cells in the TGF-*β*1-immobilized PLGA-gelatin scaffold. *Stem Cell Reviews*.

[34] Han X., Liu M., Chen D., Yan Y., Liu H., Hu W. (2019). Identification of microRNA-148a-3p with a role in transcriptional regulation of TGF-*β*2 and its relationship with antler cell proliferation. *International Journal of Agriculture And Biology*.

[35] Suttie J. M., Fennessy P. F., Gluckman P. D., Corson I. D. (1988). Elevated plasma IGF 1levels in stags prevented from growing antlers. *Endocrinology*.

[36] Russo V. C., Gluckman P. D., Feldman E. L., Werther G. A. (2005). The insulin-like growth factor system and its pleiotropic functions in brain. *Endocrine Reviews*.

[37] Vai M., Brambilla L., Orlandi I. (2000). Improved secretion of native human insulin-like growth factor 1 from gas1 mutant Saccharomyces cerevisiae cells. *Applied and Environmental Microbiology*.

[38] Hu W., Meng X., Lu T. (2013). MicroRNA-1 inhibits the proliferation of Chinese sika deer-derived cartilage cells by binding to the 3'-untranslated region of IGF-1. *Molecular Medicine Reports*.

[39] Cavallaro U., Tenan M., Castelli V. (2001). Response of bovine endothelial cells to FGF-2 and VEGF is dependent on their site of origin: relevance to the regulation of angiogenesis. *The Biochemist*.

[40] Hua Z., Lv Q., Ye W. (2006). miRNA-directed regulation of VEGF and other angiogenic factors under hypoxia. *PLoS One*.

[41] Roskoski R. (2007). Vascular endothelial growth factor (VEGF) signaling in tumor progression. *Crit Rev- oncol Hematol*.

[42] Clark D. E., Lord E. A., Suttie J. M. (2006). Expression of VEGF and pleiotrophin in deer antler. *The Anatomical Record Part A*.

[43] Mcleod D. S., Taomoto M., Cao J., Zhu Z., Witte L., Lutty G. A. (2002). Localization of VEGF receptor-2 (KDR/Flk-1) and effects of blocking it in oxygen-induced retinopathy. *Investigative Ophthalmology & Visual Science*.

[44] Dvorak H. F., Brown L. F., Dvorak A. M., Detmar M. (1995). Vascular permeability factor/vascular endothelial growth factor, microvascular hyperpermeability, and angiogenesis. *The American Journal of Pathology*.

[45] Brown L. F., Detmar M., Claffey K. (1997). Vascular permeability factor/vascular endothelial growth factor: a multifunctional angiogenic cytokine. *Regulation of Angiogenesis*.

[46] Lu L., Ting L., Li M. (2014). The transcriptional regulation of VEGF by MiRNA-93-5p and its relationship with the proliferation of sika deer antler cells. *Journal of Northeast Forestry University*.

RETRACTED

[47] Liu M., Han X., Cui D., Yan Y., Lu L., Hu W. (2019). Post-transcriptional regulation of miRNA-15a and miRNA-15b on VEGFR gene and deer antler cell proliferation. *Turkish Journal of Biochemistry*.

[48] Nieto-Diaz M., Pita-Thomas D. W., Munoz-Galdeano T. (2012). Deer antler innervation and regeneration. *Frontiers in Bioscience*.

[49] Moustakas A., Pardali K., Gaal A., Heldin C. H. (2002). Mechanisms of TGF-beta signaling in regulation of cell growth and differentiation. *Immunology Letters*.

[50] Ma L., Yang Z. Q., Ding J. L., Liu S., Guo B., Yue Z. P. (2019). Function and regulation of transforming growth factor *β*1 signalling in antler chondrocyte proliferation and differentiation. *Cell Proliferation*.

[51] Shen J., Li S., Chen D. (2014). TGF-*β* signaling and the development of osteo-arthritis. *Bone Res.*.

[52] Geiser A. G., Zeng Q. Q., Sato M., Helvering L. M., Hirano T., Turner C. H. (1998). Decreased bone mass and bone elasticity in mice lacking the transforming growth factor-beta1 gene. *Bone*.

[53] Yan Y., Chen D., Han X., Liu M., Hu W. (2020). miRNA-19a and miRNA-19b regulate proliferation of antler cells by targeting TGFBR2. *Mamm Res*.

[54] Hongyun L. (2019). *A preliminary study on the regulatory effect of miRNA-18a and miRNA-106b on the Smad family of sika deer*.

[55] Sun M., Kraus W. L. (2015). From discovery to function: the expanding roles of long noncoding RNAs in physiology and disease. *Endocrine Reviews*.

[56] Mercer T. R., Mattick J. S. (2013). Structure and function of long noncoding RNAs in epigenetic regulation. *Nature Structural & Molecular Biology*.

[57] Wilusz J. E., Sunwoo H., Spector D. L. (2009). Long noncoding RNAs: functional surprises from the RNA world. *Genes & Development*.

[58] Rinn J. L., Chang H. Y. (2012). Genome regulation by long noncoding RNAs. *Annual Review of Biochemistry*.

[59] Chuo D., Liu F., Chen Y., Yin M. (2019). lncRNA MIR503HG is downregulated in Han Chinese with colorectal cancer and inhibits cell migration and invasion mediated by TGF-*β*2. *Gene*.

[60] Chen D. Y., Jiang R. F., Li Y. J., Liu M. X., Wu L., Hu W. (2020). Screening and functional identification of lncRNAs in antler mesenchymal and cartilage tissues using high-throughput sequencing. *Scientific Reports*.

[61] Han R., Han L., Wang S., Li H. (2020). Whole transcriptome analysis of mesenchyme tissue in sika deer antler revealed the CeRNAs regulatory network associated with antler development. *Frontiers in Genetics*.

[62] Landete-Castillejos T., Kierdorf H., Gomez S. (2019). Antlers - evolution, development, structure, composition, and biomechanics of an outstanding type of bone. *Bone*.

